The article "Identification of Atrial Fibrillation-Related lncRNA Based on Bioinformatic Analysis" was retracted in 2023. Reasons: suspected computer-generated content; unreliable results or conclusions; concerns about the data; concerns about the results or conclusions.

# Identification of Atrial Fibrillation-Related lncRNA Based on Bioinformatic Analysis

**DOI:** 10.1155/2022/8307975

**Published:** 2022-02-04

**Authors:** Liangzhen Xie, GuanShen Huang, Mingjian Gao, Jianming Huang, Hai Li, Hao Xia, Xiuting Xiang, Saizhu Wu, Yunjun Ruan

**Affiliations:** ^1^Nanfang Hospital, Southern Medical University, Guangzhou, Guangdong 510515, China; ^2^Huazhong University of Science and Technology Union Shenzhen Hospital, Shenzhen, Guangdong 518000, China

## Abstract

**Background:**

Atrial fibrillation (AF) is the most common arrhythmia in the world. Long noncoding RNA (lncRNA) has been found to play an important role in cardiovascular diseases including heart failure, myocardial infarction, and atherosclerosis. However, the role of lncRNA in AF has rarely been studied. The purpose of this study is to identify the expression profile of lncRNA in AF patients, explore the function of lncRNA in AF, and provide a potential scientific basis for the treatment of AF in the future.

**Methods:**

The lncRNA and mRNA expression profiles were obtained from the atrial appendage samples of GSE31821, GSE411774, GSE79768, and GSE115574 in the Gene Expression Omnibus (GEO) database. Functional analysis was performed via Gene Ontology (GO), Kyoto Encyclopedia of Genes and Genomes (KEGG), and Gene Set Variation Analysis (GSVA). The “CIBERSORT” R kit was used to analyze 22 immune cell infiltrates in AF and sinus rhythm (SR) patients. The “CORRPLOT” R package was used to analyze the immune correlation between lncRNA and immune cells.

**Results:**

A total of 6 differentially expressed lncRNAs and 45 differentially expressed mRNAs were identified in the AF and SR groups. GO, KEGG, and GSVA results showed that abnormally expressed lncRNAs were involved in signaling pathways related to the atrium, including the Toll-like receptor signaling pathway and calcium signaling pathway. Immune cell infiltration analysis revealed that native B cells, follicular helper T cells, and resting dendritic cells may be involved in the AF process. In addition, LINC00844 was negatively correlated with resting dendritic cells.

**Conclusion:**

The expression profile of lncRNA in AF patients was different from that in normal controls. The physiological functions of these differentially expressed lncRNAs may be related to the pathogenesis of AF, which provide a scientific basis for the prognosis and treatment of patients with AF.

## 1. Introduction

Atrial fibrillation (AF) often coexists with arterial hypertension [1]. Generally, AF is positively correlated with age [2]. Elderly patients are prone to suffer from cardiovascular disease, which is often the main cause of AF [3]. However, since the pathophysiological mechanisms of AF are not yet clear, the available treatment methods are limited [4], which leads to a great public health and economic burden. Furthermore, the infiltration of immune cells regulates the inflammatory response of heart tissue, which is related to AF [5]. The cellular components of the immune system play a significant role in the development and persistence of AF [6]. In view of this, the identification of new biomarkers that affect the development of AF is essential for understanding and preventing the disease in the future.

The article "Identification of Atrial Fibrillation-Related lncRNA Based on Bioinformatic Analysis" was retracted in 2023. Reasons: suspected computer-generated content; unreliable results or conclusions; concerns about the data; concerns about the results or conclusions.

With the development of high-throughput sequencing and molecular biology, it is possible to explore the pathogenesis of diseases at the molecular level [7]. Many studies have proved that noncoding RNA is a regulator of heart disease [8]. For example, microRNA (miRNAs) is a small noncoding RNA that has an interesting connection with AF [9]. In addition, long noncoding RNA (lncRNA) is a novel noncoding RNA with a length of more than 200 nt [10]. For the moment, growing literatures report that lncRNAs can become new biomarkers for disease diagnosis and prognosis [11]. There were 389 differentially expressed lncRNAs in cardiac fibrotic and distal ventricular tissue of myocardial infarction [12]. lncRNA GAS5 protected cardiomyocytes from hypoxia injury [13]. Similarly, there is also evidence that lncRNA is abnormally expressed in ventricular septal defect, heart failure, and other heart diseases [14]. Unfortunately, to the best of our knowledge, no one has attempted to study the relationship between the expression of lncRNA and AF, and its potential pathway is still unknown.

In this study, we proposed to identify potential key lncRNAs of AF using bioinformatic methods through Gene Expression Omnibus (GEO) and analyze its expression, function, and interaction.

## 2. Methods

### 2.1. Microarray Data

The original files of 4 registered microarray datasets were downloaded from the NCBI Gene Expression Omnibus (GEO) database (https://www.ncbi.nlm.nih.gov/geo/), including GSE31821, GSE411774, GSSE79768, and GSE115574 (Table 1). All data are from Affymetrix Human Genome U133 Plus 2.0 Array (HGU133_Plus_2). We selected human atrial appendage samples from subjects with AF and sinus rhythm (SR) in each group and finally selected 78 AF and 51 SR samples for subsequent analysis.

### 2.2. Data Processing

Process the sequence matrix file through Perl software, and convert the gene probe ID into the gene symbol code. After merging all microarray data, the batch effects were adjusted by the “combat” function of the “sva” package of R software using the empirical Bayes framework. According to the literature [15], Affymetrix microarray probes were reannotated with lncRNAs, and 3873 lncRNAs were obtained. After the probes annotated to the same lncRNA were combined, 3005 lncRNAs were finally obtained. Finally, the expression value according to the “normalize Between Arrays” function in the “limma” package of R software was normalized, so that the expression value has a similar distribution in a group of arrays.

The article "Identification of Atrial Fibrillation-Related lncRNA Based on Bioinformatic Analysis" was retracted in 2023. Reasons: suspected computer-generated content; unreliable results or conclusions; concerns about the data; concerns about the results or conclusions.

### 2.3. Identification of Differentially Expressed lncRNAs and mRNAs

In order to evaluate the differential expression, the standard error was adjusted by using the “limma” package of R software, linear model fitting, and a simple empirical Bayes model [16]. For each comparison of each gene, a moderate *t* statistic and the logarithm of differential expression were calculated. We then adopted the Benjamini and Hochberg (BH) method to adjust the *P* value to reduce false-positive errors. Differentially expressed lncRNAs and mRNAs were identified between the AF and SR samples through fold change (FC) and *P* value filtering (︳log2FC︳>0.58 and *P* < 0.05), which were visualized as volcano plots and heat map plots.

### 2.4. Biomathematical Analyses

The preliminary differentially lncRNA-mRNA network and differentially lncRNA-functional enrichment pathway were built using Cytoscape software (version 3.6.1). The related genes in lncRNA regulatory network were performed for GO and pathway enrichment analyses using GO (http://www.geneontology.org/) and the Database for Annotation, Visualization, and Integrated Discovery (DAVID; https://david.ncifcrf.gov/).

### 2.5. Gene Set Variation Analysis (GSVA)

GSVA is a pathway enrichment method used to estimate the changes in pathway activity in a sample population. The R software package of GSVA was downloaded at http://www.bioconductor.org. We predicted the pathway in AF and SR states based on the signal value of the gene and the pathway where the gene is located. The enriched score value of each sample was predicted by the signal value of the gene, and the pathway with differential enrichment in the two groups was obtained. The screening standard *P* < 0.05, and the FDR < 0.05.

### 2.6. Immunoinfiltration Analysis

In order to better understand the situation of infiltrating immune cells in the AF and SR groups, we used the CIBERSORT algorithm to calculate the relative proportion of infiltrating immune cells. Then, the Wilcoxon test was used to compare the constituent fractions of infiltrating immune cells in the AF group and the SR group, in which *P* value < 0.05 was significant. In addition, Pearson correlation analysis was performed to find out the relationship between each ideal lncRNA and significantly infiltrated immune cells.

The article "Identification of Atrial Fibrillation-Related lncRNA Based on Bioinformatic Analysis" was retracted in 2023. Reasons: suspected computer-generated content; unreliable results or conclusions; concerns about the data; concerns about the results or conclusions.

### 2.7. Immune Correlation Analysis of Differential lncRNA

We used the Pearson coefficient test to test the correlation of immune infiltrating cells. The Spearman coefficient test was used to test the correlation between the proportion of immune cells and differential lncRNAs. Finally, with the help of “corrplot” R packages, we drew a correlation diagram to report the immune correlation between lncRNA and immune cells. *P* value < 0.05 was considered as a statistically significant threshold.

### 2.8. Statistical Analysis

R software 3.6.1 was used for statistical analysis. ︳log2FC︳>0.58 and *P* < 0.05 were the filtering criteria for differential genes. Pearson correlation coefficient was performed to determine the gene coexpression. Statistical significance was determined at *P* < 0.05.

## 3. Results

### 3.1. Identification of Differentially lncRNA and mRNA Expression Profile

The analysis process of this study is shown in Figure 1. In total, 3,005 lncRNAs were identified by GSE31821, GSE411774, GSSE79768, and GSE115574 microarray datasets. A total of 6 lncRNAs were differentially expressed between the SR group and the AF group (log2FC > 0.58 and *P* < 0.05), compared with SR groups: 4 lncRNAs were upregulated and 2 were downregulated in AF groups (Figures 2(a) and 2(b)). In addition, we also found 45 differentially expressed mRNAs, of which 31 mRNAs were downregulated and 14 were upregulated in AR groups compared with SR groups (Figures 3(a) and 3(b)).

### 3.2. Identification of lncRNA-mRNA Regulatory Coexpression Network

By analyzing the correlation between differentially expressed lncRNAs and mRNAs, the regulatory network between lncRNAs and mRNAs was constructed. As shown in Figure 4, the regulatory network was complicated. For instance, RP11-432J24.5 had a negative regulatory relationship with TCEAL2, TNNI1, and SFRP5, and a positive regulatory relationship with RPL3L, which indicated that the roles of these differentially expressed lncRNAs are diverse in patients with AF.

### 3.3. Gene Ontology Functions and Pathway Enrichment Analysis

Functional enrichment analysis indicated that the related genes in lncRNA regulatory network were mainly involved in GO terms, including “transmembrane signaling receptor activity,” “multicellular organism development,” “G-protein coupled receptor activity,” “protein binding,” and “plasma membrane” (Figure 5(a)). Additionally, KEGG pathway enrichment analysis for the related genes in lncRNA regulatory network was performed to further study biological function. Briefly, these genes were mainly participated in “thyroid hormone signaling pathway,” “adrenergic signaling in cardiomyocytes,” “insulin resistance,” “cAMP signaling pathway,” and “cardiac muscle contraction” (Figure 5(b)). These results suggest that differential lncRNAs play different physiological functions and participate in the regulation of AF.

The article "Identification of Atrial Fibrillation-Related lncRNA Based on Bioinformatic Analysis" was retracted in 2023. Reasons: suspected computer-generated content; unreliable results or conclusions; concerns about the data; concerns about the results or conclusions.

### 3.4. GSVA Analysis

The GSVA was used to figure out the dynamics of biological pathways and processes. We found that the AF group were enriched in GO term, such as “t cell homeostasis,” “positive regulation of protein autophosphorylation,” “interleukin7-mediated signaling pathway,” and “response to hyperoxia” (Figure 6(a)). For pathway, “thyroid cancer,” “Toll-like receptor signaling pathway,”, “RNA degradation,” and other cancer pathways were highly enriched in the AF group, compared with the SR group (Figure 6(b)). Furthermore, we then analyzed the correlation between these differential functions and pathways and differential lncRNAs. As shown in Figure 6(c), LINC00844 positively regulated “GO_ATPASE_ACTIVATOR_ACTIVITY” and negatively regulated “GO_POSITIVE_REGULATION_OF_CALCIUM_ION_TRANSPORT,” “GO_POSITIVE_REGULATION_OF_CALCIUM_ION_TRANSPORT,” “GO_CORONARY_VASCULATURE_DEVELOPMENT,” “GO_POSITIVE_REGULATION_OF_CARDIAC_MUSCLE_CELL_DIFFERENTIATION,” “GO_ACTIN_FILAMENT,” and “GO_ACTIN_BINDING.” RP11-432J24.5 and UNC5B-AS1 together negatively regulated “GO_SOMITE_DEVELOPMENT.”

### 3.5. The Immune Cell Infiltration Landscape in AF and SR

In order to further explore the composition of immune cells in AF and SR groups, we investigated the immune cell infiltration landscape by using the CIBERSORT algorithm. Reasonably, the results showed that there was a significant difference in the proportion of tumor-infiltrating immune cells between the AF group and the SR group (Figure 7(a)). We then constructed a violin chart to compare the difference in immune cell infiltration between the AF group and the SR group. As shown in the figure, compared with SR groups, “B cells native” (*P* = 0.019) was highly expressed in AR groups, whereas “T cells follicular helper” (*P* = 0.049) and “dendritic cells resting” (*P* = 0.041) were reduced in AR groups (Figure 7(b)). The correlation of 22 types of immune cells revealed that native B cells and follicular helper T cells were all positively related to CD8+ T cells (*r* = 0.1 and *r* = 0.04, respectively) and resting dendritic cells were positively related to follicular helper T cells (*r* = 0.05), whereas native B cells were negatively related to follicular helper T cells and resting dendritic cells (*r* = −0.14 and *r* = −0.06, respectively), and resting dendritic cells were negatively related to CD8+ T cells (*r* = −0.06) (Figure 7(c)). There is a significant difference in immune cell infiltration between heart tissue in patients with AF and SR groups. Therefore, B cells, dendritic cells, CD8+ T cells, and follicular helper T cells may be potential core immune cells, involved in stimulating the progression of AF.

The article "Identification of Atrial Fibrillation-Related lncRNA Based on Bioinformatic Analysis" was retracted in 2023. Reasons: suspected computer-generated content; unreliable results or conclusions; concerns about the data; concerns about the results or conclusions.

### 3.6. Correlation Analysis between Differential lncRNA and Differential Immune Cells

After the correlation analysis, only LINC00844 had a statistically significant relationship with immune cells. The scatter diagrams displayed the correlation between lncRNA expression and immune cells. The results showed that LINC00844 was negatively associated with marker genes of dendritic cells resting (*R* = −0.28, *P* = 0.0014) (Figure 8). The above data showed that LINC00844 inhibits immune response by affecting dendritic cells in AF.

## 4. Discussion

AF is the main cause of ischemic stroke, accompanied by arrhythmia [17]. Currently, the prevalence of AF is increasing, but the effects of available treatments are limited [18]. Understanding the molecular mechanism and pathogenesis signature of AF is often of great significance to the treatment of the disease [19]. The vigorous development of microarray technology provided opportunities for the treatment of AF. In the present research, we downloaded the AF microarray data from the GEO database and found that there were differentially expressed lncRNAs in the atrial tissues between AF patients and healthy patients. Simultaneously, compared with SR groups, 31 mRNAs were downregulated and 14 mRNAs were upregulated in AF groups. Therefore, we constructed the lncRNA-mRNA interaction network. Afterwards, through gene enrichment analysis and GSVA analysis, we found that differential lncRNA can affect the biological functions of atrial hypertrophy, myocarditis, and immune cells in AF patients. Finally, we identified a negative correlation between LINC00844 and dendritic cells resting.

With the rapid development of RNA sequencing technology, more and more noncoding RNAs have been discovered. One of the new molecules called lncRNA has become a famous molecule in biological research [20]. According to reports, from cancer to cardiovascular disease, lncRNA dysfunction was associated with a wide range of disease phenotypes [21, 22]. A recent study showed that braveheart is a mouse heart-related lncRNA, which was identified as a key regulator of cardiovascular commitment [23]. In addition, some studies have found that MIAT is a type of lncRNA that increases the risk of myocardial infarction [24]. In the current study, we identified 6 differentially expressed lncRNAs between AF groups and SR groups, among which 2 lncRNAs were downregulated and 4 lncRNAs were upregulated. Similarly, in other similar reports, lncRNA PVT1 increased in atrial muscle tissue of patients with AF, resulting in atrial fibroblast proliferation [25]. As other reports have stated, abnormally expressed lncRNA could cause a variety of diseases at the level of gene transcription or regulatory functions and pathways [26]. Based on the above results, we speculated that these abnormally lncRNAs may play an important role in AF patients. lncRNA regulates gene expression by participating in regulating the transcription and translation of genes [27]. Moreover, lncRNA affects the characterization of diseases by regulating the expression of mRNA [28]. Based on the GEO database, we screened out differential expressed lncRNAs and mRNAs and performed correlation analysis to construct a regulatory network of differential lncRNAs-mRNAs via bioinformatic analysis. Then, we conducted GO and KEGG analysis on the differential genes in the regulatory network. GO enrichment analysis showed that the differential expression of lncRNA is mainly involved in the metabolic process, catabolism process, and biosynthesis process in the biological process. Furthermore, lncRNA LncHrt has been reported to maintain cardiac metabolic homeostasis and cardiac function by regulating the LKB1-AMPK signaling pathway [29]. However, in our study, KEGG analysis manifested that most enriched pathways were related to adrenergic signaling in cardiomyocytes, the thyroid hormone signaling pathway, and cardiac muscle contraction. There is increasing evidence that the main mechanism of arrhythmia may depend on cardiology and adrenergic stress [30]. Reports showed that patients with extremely low levels of thyroid-stimulating hormone are at higher risk of death from coronary heart disease and AF [31]. These evidences indicated that differentially expressed lncRNA may affect the occurrence, progression, and maintenance of AF by accommodating the expression of its corresponding mRNA. In addition to conventional GO and KEGG analysis, we also used GSVA for the first time to estimate changes in pathway activity in a sample population [32]. Through GSVA analysis, we found that the occurrence of AF is mainly related to changes in the Toll-like receptor signaling pathway and the interleukin 7-mediated signaling pathway. Finally, we found that differential lncRNA is mainly involved in the calcium signaling pathway. Increasing evidences show that atrial tachyarrhythmia causes atrial hypertrophy by activating the Ca^2+^ signaling pathway, which thereby leads to structural remodeling of the atria [33–35]. These indicated that these signaling pathways might be involved in the initiation and development of AF and differentially expressed lncRNAs might take part in the pathogenesis of AF.

The article "Identification of Atrial Fibrillation-Related lncRNA Based on Bioinformatic Analysis" was retracted in 2023. Reasons: suspected computer-generated content; unreliable results or conclusions; concerns about the data; concerns about the results or conclusions.

Immune responses are significantly related to the recurrence and maintenance of AF [36]. All kinds of immune cells, including innate immune cells and adaptive immune cells, infiltrated the atrium and interacted with the atrial cardiomyocytes to regulate the cardiac microenvironment [37]. However, regarding the AF, immune infiltration analyses are not abundant, thus with the help of CIBERSORT, we evaluated the expression level of 22 kinds of immune cells in AF. The results showed that “B cells native” were upregulated, and “dendritic cells resting” and “T cells follicular helper” were downregulated in AF. Recent studies have confirmed that immune cells are of great significance to the onset time of AF and the remodeling of the atrium [38]. We likewise analyzed the correlation between differential lncRNA and immune cells, which was found that LINC00844 was negatively correlated with resting dendritic cells. Similarly, some lncRNAs can suppress CD8+ T cells to enhance drug resistance [39]. Collectively, the above results indicated that differentially expressed lncRNA affects AF through immune and inflammatory signaling pathways.

## 5. Conclusions

Our study integrated data with a relatively larger sample size from multiple GEO datasets and identified 6 potential crucial genes (RP11-532N4.2, RP3-332B22.1, RP11-557H15.4, RP11-432J24.5, UNC5B-AS1, and LINC00844). In addition, 45 differential mRNAs were identified and an interaction map was established between differential mRNAs and lncRNAs. Then, we analyzed the differential lncRNAs in the network by using bioinformatic analyses. Besides, we also analyzed the immune cell infiltration landscape between AF and SR. Furthermore, attention should be paid to the relationship between linc00844 and dendritic cells resting, which may be a new direction of AR research in the future. Our research results may provide new biomarkers and effective therapeutic targets for the diagnosis and treatment of AF.

## 6. Limitations

Our study has several limitations. First, although this is a multiomics integrated analysis, those external clinical features were not used in our study. Secondly, we did not verify these differential lncRNAs by constructing relevant animal models.

## Figures and Tables

**Figure 1:** Flow chart of the study.

**Figure 2:** Expression profile of lncRNA in AF and SR. (a) The heat map visualized changes in lncRNA expression using hierarchical clustering analysis. (b) The volcano plot showed the differentially expressed lncRNAs between different groups (the SR and AF patients). Green represented downregulated lncRNAs, and red represented upregulated lncRNAs.

The article "Identification of Atrial Fibrillation-Related lncRNA Based on Bioinformatic Analysis" was retracted in 2023. Reasons: suspected computer-generated content; unreliable results or conclusions; concerns about the data; concerns about the results or conclusions.

**Figure 3:** Expression profile of mRNA in AF. (a) The heat map visualized changes in mRNA expression using hierarchical clustering analysis. (b) The volcano plot showed the differentially expressed mRNAs between different groups (the SR and AF patients). Green represented downregulated lncRNAs, and red represented upregulated lncRNAs.

**Figure 4:** The construction of coexpression network of lncRNA-mRNA using Cytoscape software. The diamond represents lncRNA, and the circular represents mRNA. The yellow represented downregulated, and purple represented upregulated.

**Figure 5:** Functional enrichment analysis of the related genes in lncRNA regulatory network. (a) GO enrichment analysis of differentially expressed mRNAs. (b) KEGG-enriched terms of differentially expressed mRNAs.

**Figure 6:** The changes of pathway activity in the sample population were analyzed by GSVA analysis. (a) The cluster heat map showed the GO terms of GSVA between AF and SR groups. (b) The cluster heat map showed the pathways of GSVA between AF and SR groups. (c) The lncRNA-pathway coexpression network. The ellipse represents mRNA, and the V represents lncRNA; blue indicated downregulated, and orange indicated upregulated; green indicated positive correlation, and purple indicated negative correlation.

**Figure 7:** The immune cell infiltration landscape in AF and SR. (a) Heat map of the infiltrating cell proportions. (b) Violin plot showed the different proportions of infiltrating cells between the AF group and the SR group. (c) Correlation matrix of immune cell proportions.

**Figure 8:** LINC00844 was negatively associated with resting dendritic cells.

**Table 1:** Characteristics of samples in the datasets of this study.

GSE series	Total	AF	SR
GSE31821	6	4	2
GSE41177	38	32	6
GSSE79768	26	14	12
GSE115574	59	28	31

## Data Availability

The datasets generated for this study can be found in the GEO database (GSE31821, GSE411774, GSSE79768, and GSE115574; https://www.ncbi.nlm.nih.gov/geo/).
